# Correlations between Intestinal Microbiota and Clinical Characteristics in Colorectal Adenoma/Carcinoma

This article has been retracted.

**DOI:** 10.1155/2022/3140070

**Published:** 2022-07-28

**Authors:** Caizhao Lin, Baolong Li, Chunyi Tu, Xiaohua Chen, Min Guo

**Affiliations:** ^1^Department of Colorectal Surgery, The First Affiliated Hospital, College of Medicine, Zhejiang University, China; ^2^Department of General Surgery, The Fifth Affiliated Hospital, Southern Medical University, Guangzhou, Guangdong, China; ^3^Department of Gastroenterology, The First Affiliated Hospital of Jinan University, Guangzhou, Guangdong Province 510630, China; ^4^Department of Biochemistry, Medical College of Shaoguan University, Shaoguan, Guangdong Province 512026, China; ^5^Department of Oncology, The Fifth Affiliated Hospital, Southern Medical University, Guangzhou, Guangdong 510515, China

## Abstract

**Background:**

Most of colorectal cancer (CRC) cases are sporadic and develop along the adenoma-carcinoma sequence. Intestinal microbial dysbiosis is involved in the development of colorectal cancer. However, there are still no absolute markers predicting the progression from adenoma to carcinoma.

**Aims:**

To investigate the characteristics of intestinal microbiota in colorectal adenoma and carcinoma patients and the correlations with clinical characteristics.

**Methods:**

Fecal samples were collected from 154 colorectal carcinoma patients (CRC group), 20 colorectal adenoma patients (AD group), and 199 healthy controls (control group). The intestinal microbiota was investigated by 16S rRNA gene sequencing.

**Results:**

Compared to the healthy controls, microbial diversity was dramatically decreased in AD/CRC. At the genus level, *Acidaminococcus* significantly decreased with the order of control-AD-CRC (*P* < 0.05). *Parvimonas*, *Peptostreptococcus*, *Prevotella*, *Butyricimonas*, *Alistipes*, and *Odoribacter* were the key genera in the network of colorectal adenoma/carcinoma-associated bacteria. Combination of the top 10 most important species, including *Butyricimonas synergistica*, *Agrobacterium larrymoorei*, *Bacteroides plebeius*, *Lachnospiraceae* bacterium feline oral taxon 001, *Clostridium scindens*, *Prevotella heparinolytica*, bacterium LD2013, *Streptococcus mutans*, *Lachnospiraceae* bacterium 19gly4, and *Eubacterium hallii*, showed the best performance in distinguishing AD patients from CRC (AUC = 85.54%, 95% CI: 78.83%-92.25%). The clinicopathologic features, including age, sex, tumor location, differentiation degree, and TNM stage, were identified to be closely linked to the intestinal microbiome in CRC.

**Conclusion:**

Several intestinal bacteria changed along the adenoma-carcinoma sequence and might be the potential markers for the diagnosis and treatment of colorectal adenoma/carcinoma. Intestinal microbiota characteristics in CRC should account for the host factors.

## 1. Introduction

Colorectal cancer (CRC) is the fourth most deadly cancer worldwide [1]. In China, CRC is the fourth most common cancer diagnosed in males and the third most common cancer diagnosed in females [2]. The etiology of CRC is associated with many factors, including genetic and environmental factors [3]. Intestinal microbiota plays an important role in the environmental factor and contributes to the development of CRC [4]. However, the specific mechanisms and functional capacity are not fully understood.

Most of the sporadic CRC develops along the adenoma-carcinoma sequence. An increasing number of studies have shown that the intestinal microbiota altered during the development along the adenoma-carcinoma sequence [5–7]. Several microbes, such as *Fusobacterium nucleatum*, *Bacteroides fragilis*, *Enterococcus faecalis*, and *Clostridium symbiosum*, have been reported in association with tumorigenesis and might be the potential biomarkers for the detection of CRC [6, 8–11]. However, the results of present studies were not consistent, possibly attributed to the differences in sampling (fecal or mucosal tissue) or processing method (RT-PCR or high-throughput analyses) or different stages of tumor or location differences between the left side and right side [9]. There are still no absolute markers predicting the progression from adenoma to carcinoma.

In this study, fecal samples from 154 colorectal carcinoma patients and 20 colorectal adenoma patients were collected. The first aim was to characterize the microbiota differences along the adenoma-carcinoma sequence based on 16S rRNA gene sequencing. It was revealed that the microbiome characteristic in AD was quite similar to that in CRC. Several intestinal bacteria changed along the adenoma-carcinoma sequence and might be the potential markers for the diagnosis and treatment of colorectal adenoma/carcinoma. The second aim was to explore the correlations between the intestinal microbiota and clinical characteristics. The clinicopathologic features, including age, sex, tumor location, differentiation degree, and TNM stage, were closely linked to the intestinal microbiome in CRC. Our findings provide more knowledge for elucidating the tumorigenesis and offer a basis for the development of more effective strategies for the clinical treatment of CRC in the future.

## 2. Methods

### 2.1. Study Population and Sampling

Participants were from outpatients who received the colonoscopy at the First Affiliated Hospital, Zhejiang University School of Medicine. All colorectal adenoma patients and colorectal cancer patients had not undergone endoscopic or surgical treatment. Exclusion criteria included patients older than 90 years of age, patients with a personal history of colorectal cancer, colorectal adenoma, and inflammatory bowel disease or a family history of colorectal cancer, and patients who had used antibiotics within two months or received chemotherapy/radiation treatments within six months. Colonoscopy was performed by experienced endoscopists. Written informed consent was obtained from all participants. From June 2020 to December 2020, fresh fecal samples (≥1 g) were collected from all participants before colonoscopy and immediately frozen at -80°C until further processing for 16S rRNA gene sequencing analysis. The clinical characteristics of the patients were recorded, including age, sex, tumor size, location, TNM stage, differentiation degree, pathological pattern, and histology. Unfortunately, we were not able to recruit healthy controls in the First Affiliated Hospital, Zhejiang University School of Medicine. Therefore, the corresponding data of control (*n* = 199) was obtained from the Kesic Dataset of a project for predicting the age based on the gut microbiota (https://www.kesci.com/home/project/5ddb6bedf41512002cebd995). The study protocol was approved by the Medical Ethics Committee of the First Affiliated Hospital, Zhejiang University School of Medicine (2017-869). In addition, all patients signed informed consent forms.

### 2.2. DNA Extraction and 16S rRNA Gene Sequencing

Total genomic DNA extraction from fecal samples was performed using a QIAamp DNA Stool Mini Kit (QIAGEN, Germany) following the manufacturer's instructions. The quality and concentration of DNA were verified with 2% agarose gel (Tanon, China) and a NanoDrop spectrophotometer (Thermo Fisher Scientific, USA).

High-throughput Illumina sequencing of the V3-V4 variable regions of the 16S rRNA gene was performed using universal primers 343F (5′-TACGGRAGGCAGCAG-3′) and 798R (5′-AGGGTATCTAATCCT-3′). The PCR reaction was carried out with 15 *μ*L of Phusion® High-Fidelity PCR Master Mix (New England Biolabs, United States), 0.2 *μ*M of forward and reverse primers, and about 10 ng template DNA. Thermal cycling consisted of initial denaturation at 98°C for 1 min, followed by 30 cycles of denaturation at 98°C for 10 s, annealing at 50°C for 30 s, and elongation at 72°C for 30 s followed by a final extension of 5 min at 72°C.

The amplicon was purified with AMPure XP beads (Beckman Coulter, USA) and subjected to a secondary PCR reaction. The final amplicon was quantified using a Qubit dsDNA assay kit (Life Technologies, USA). A sequencing library was generated using the TruSeq® DNA PCR-Free Sample Preparation Kit (Illumina, USA) following the manufacturer's recommendations and assessed on the Qubit^@^ 2.0 Fluorometer (Thermo Fisher Scientific, USA) and Agilent Bioanalyzer 2100 system (Agilent Technologies, USA). The library was sequenced on an Illumina NovaSeq platform, and 250 bp paired-end reads were generated.

### 2.3. Bioinformatics and Statistical Analysis

The FASTQ files were processed using QIIME (V1.9.1, http://qiime.org/scripts/split_libraries_fastq.html). Paired-end reads were merged using FLASH (V1.2.7, http://ccb.jhu.edu/software/FLASH/). Quality filtering on the raw tags was performed under specific filtering conditions to obtain high-quality clean tags. The effective tags were obtained by detected chimera sequences, and the chimera sequences were removed using the UCHIME algorithm (UCHIME algorithm version 10.0, http://www.drive5.com/usearch/manual/uchime_algo.html) based on the reference database (SILVA database version 123, https://www.arb-silva.de/). Sequences with 97% sequence homology were assigned to the same operational taxonomic units (OTUs) by using UPARSE software (version 7.0.1001, http://www.drive5.com/uparse/). The representative sequence for each OTU was screened for further annotation. All representative reads were annotated and blasted against the SILVA database (version 123, http://www.arb-silva.de/) using the RDP classifier (confidence threshold was 70%). OTU abundance information was normalized using a standard of sequence number corresponding to the sample with the least sequences.

Alpha diversity and beta diversity analyses were performed by using QIIME (version 1.9.1). Alpha diversity was applied in analyzing complexity of species diversity for samples. The community richness and diversity were described by the Chao index and Shannon index, respectively. Beta diversity analysis was used to evaluate comparisons between groups among samples and assessed by nonmetric multidimensional scaling (NMDS) analysis and principal coordinate analysis (PCoA) by using a weighted UniFrac distance matrix. Linear discriminant analysis (LDA) effect size [12] was used to identify differentially abundant bacterial taxa associated with groups of participants. The LDA value threshold was set at 4. The *t*-test and Wilcox test were employed to assess the significance by using QIIME (version 1.9.0).

## 3. Results

### 3.1. Characteristics of Subjects

A total of 373 participants, including 154 CRC patients (mean age of 65.81 ± 10.98 years, 63.64% male), 20 AD patients (mean age of 64.35 ± 12.89 years, 75.00% male), and 199 healthy controls (mean age of 59.48 ± 3.20 years, 58.29% male), were enrolled in this study. The clinical characteristics of the patients are shown in Table 1. The mean size of carcinoma was 4.55 ± 2.18 mm, and most of the tumors were found in the left colon (75.97%). In the CRC group, the differentiation degree concentrated in the moderate degree (75.32%) and mainly tubular adenocarcinoma (85.06%).

### 3.2. Summarization of 16S rRNA Gene Sequencing Results

A total of 2,668 OTUs were generated from 164 patients' samples. The Venn diagram showed that 1,323 OTUs were shared between AD and CRC, while 113 unique OTUs existed in AD and 1232 unique OTUs existed in CRC (Figure 1(a)). The rarefaction curve and species accumulation boxplot are shown in Figures 1(b) and 1(c). The value of Good's coverage for each group was over 99.8% (Figure 1(d)). No significant difference in alpha diversity was observed between AD and CRC groups (*P* = 0.95 for the Chao index, Figure 1(e); *P* = 0.74 for the Shannon index, Figure 1(f)). A mild separation between AD and CRC was observed, and no significant difference in microbiota composition was detected by PCoA (*Pr*(>*F*) = 0.33 for weighted UniFrac distance, Figure 1(g)). NMDS analysis also revealed that the microbiota composition between the two groups was similar; samples from AD and CRC mostly overlapped with one another (stress = 0.202 > 0.2, Figure 1(h)). The analysis of beta diversity revealed that fecal microbial communities between AD and CRC were not distinct from each other (*P* = 0.88 for weighted UniFrac distance, Figure 1(i)). However, there was more dispersion in control samples than in AD/CRC samples in both the PCoA and NMDS plots (stress = 0.123 < 0.2, Figures 1(j) and 1(k)), suggesting that the fecal microbial communities between control and AD/CRC were different.

### 3.3. Specific Bacterial Taxa Associated with Colorectal Adenoma/Carcinoma and Potential Diagnostic Biomarker

The bacterial community from 154 CRC and 20 AD patients' fecal samples was classified into 28 phyla, 45 classes, 99 orders, 178 families, 423 genera, and 461 species. At the genus level, the intestinal microbiota was dominated by *Bacteroides* (30.75%), *Prevotella* (14.03%), and *Faecalibacterium* (5.51%) in control (Figure 2(a)). The dominant genera in CRC were *Bacteroides* (25.92%), *Faecalibacterium* (6.39%), and *Fusobacterium* (3.38%), while the dominant genera in AD were *Bacteroides* (25.92%), *Faecalibacterium* (6.39%), and *Blautia* (4.08%) (Figure 2(a)).

The significant analysis based on the Wilcox test showed that 115 genera of intestinal microbiota in AD patients were distinct from those in controls. Correspondingly, there were 134 genera significantly different in CRC patients compared with control (Figure 3(a)). Besides, there were 4 genera significantly different among the three groups, namely, *Acidaminococcus*, *Alloprevotella*, *Mycoplasma*, and *Sphingobacterium* (Figure 3(b)). Notably, the relative abundance of *Acidaminococcus* was decreased with the order of control-AD-CRC. LEfSe analysis was used to identify the specific taxa associated with CRC. Only one family (Prevotellaceae) is enriched in CRC (Figure 3(c)). *Parvimonas*, *Peptostreptococcus*, *Prevotella*, *Butyricimonas*, *Alistipes*, and *Odoribacter* were key genera in the network of colorectal adenoma/carcinoma-associated bacteria (Figure 3(d)). Furthermore, random forest analysis suggested that a combination of the top 10 species showed the best performance in distinguishing AD patients from CRC patients (AUC = 85.54%, 95% CI: 78.83%-92.25%, Figure 3(e)). Mean Decrease Gini (MDG) and Mean Decrease Accuracy (MDA) coefficients were used to rank the importance of the variables from random forest algorithm results (Figures 3(f) and 3(g)). The 10 most important species were *Butyricimonas synergistica*, *Agrobacterium larrymoorei*, *Bacteroides plebeius*, *Lachnospiraceae* bacterium feline oral taxon 001, *Clostridium scindens*, *Prevotella heparinolytica*, bacterium LD2013, *Streptococcus mutans*, *Lachnospiraceae* bacterium 19gly4, and *Eubacterium hallii*.

### 3.4. Association between Fecal Microbiota and CRC Clinical Characteristics

To explore the correlations between intestinal microbiota and clinical characteristics, we created the correlation heatmap according to the different clinicopathologic features of CRC patients. As shown in Figure 4(a), 154 patients were divided into two groups according to their age: 13 CRC patients were younger than 50 years old and 141 patients were older than 50 years old, and 15 bacterial species were higher and another 15 bacterial species were significantly lower in the old patients than in the young patients. Additionally, 1 phylum (Firmicutes, *P* < 0.05, data not shown) dramatically decreased in the old patients compared to the young patients. Stratified by sex, a heatmap was created to summarize the association between the microbiome and sex (Figure 4(b)), and 5 bacterial species increased in female patients including *Prevotella* sp. Marseille-P2931, *Clostridium colinum*, *Bifidobacterium pseudocatenulatum*, *Gordonibacter* sp. Marseille-P2775, and *Saccharibacteria bacterium* UB2523. The other 11 bacterial species are significantly enriched in male patients (Figure 4(b)).  Figure 4(c) shows the association results stratified by tumor location. The microbiome was different between the patients with the tumor in the left and right colon, in which 17 bacterial species were found obviously changed (7 up and 10 down, left vs. right). Interestingly, the relative abundance of *Bacteroides cellulosilyticus* was significantly increased with the order of differentiation degree in poor-moderate-well (*P* < 0.05, data not shown). Furthermore, we compared the relationship between microbiota and tumor stages in CRC (I-II vs. III-IV). The relative abundances of 9 bacterial species, including *Porphyromonas uenonis*, *Clostridium colinum*, *Proteiniphilum* sp., *Selenomonas ruminantium*, *Gordonibacter* sp. Marseille-P2775, *Akkermansia muciniphila*, *Rikenella microfusus*, *Dialister pneumosintes*, and *Weissella cibaria*, were significantly higher in the TNM stage III/IV group than in the TNM stage I/II group (Figure 4(d)).

## 4. Discussion

In summary, our study identified colorectal adenoma/carcinoma-associated microbes in AD/CRC patients compared with controls. CRC-associated bacteria altered with the colorectal adenoma-carcinoma sequence. Combining with the ten genera of colorectal adenoma/carcinoma-associated bacteria can effectively distinguish AD and CRC patients. The host clinicopathologic features, such as age, sex, tumor location, differentiation degree, and TNM stage, were closely linked to the intestinal microbiome in CRC. Disease outcomes of CRC should account for microbiota characteristics and host factors in the future.

In this study, the intestinal microbiota in AD or CRC patients was distinct from that in healthy controls, which was primarily attributed to a decrease in bacterial diversity. However, the species richness and community diversity were not markedly altered between AD and CRC. There was only family Prevotellaceae that was significantly enriched in CRC compared to AD by LEfSe analysis. The intestinal microbiome of CRC was dominated by the genus of *Bacteroides*, *Faecalibacterium*, and *Fusobacterium*, which was consistent with some previous studies [12–14]. In AD, the dominant genera were *Bacteroides*, *Faecalibacterium*, and *Blautia*. *Blautia* was a butyrate-producing bacterium that is enriched in the human gut. Recently, it was found that *Blautia* was the special gut microbe significantly associated with visceral fat accumulation in Japanese adults [15].

In this study, *Acidaminococcus*, *Alloprevotella*, *Mycoplasma*, and *Sphingobacterium* were identified to be significantly altered among the three groups, in which *Acidaminococcus* was decreased with the order of control-AD-CRC. However, the enrichment of *Acidaminococcus intestini* was found to be higher in carcinomas than in controls and negatively correlated with the dietary indices (red meat and serum ferritin) in previous studies [6]. These discrepant results may be due to the differences between the study populations. Furthermore, we also analyzed the interplay between CRC- and AD-associated bacterial genera. In the network analysis, we observed the close relationship between colorectal adenoma/carcinoma and oral pathogens, such as *Parvimonas* and *Peptostreptococcus*. These bacteria were reported to be enriched in tumor tissues or feces of individuals with CRC or adenomas and involved in the carcinogenesis of the CRC [9, 16, 17]. Our results provided additional evidence that oral periodontopathic bacteria played an important role in tumorigenesis of CRC. Additionally, *Prevotella*, *Alistipes*, *Butyricimonas*, and Odoribacter were also identified as the colorectal adenoma/carcinoma-associated bacteria, which was consistent with previous research [6, 9, 18, 19].

Our results showed that the combination of the 10 species can distinguish colorectal adenoma from CRC, namely, *Butyricimonas synergistica*, *Agrobacterium larrymoorei*, *Bacteroides plebeius*, *Lachnospiraceae* bacterium feline oral taxon 001, *Clostridium scindens*, *Prevotella heparinolytica*, bacterium LD2013, *Streptococcus mutans*, *Lachnospiraceae* bacterium 19gly4, and *Eubacterium hallii*. These special species have been identified as the CRC-associated bacteria, such as genera *Bacteroides*, *Prevotella*, *Clostridium*, and *Streptococcus* [6, 13]. These results suggested that these 10 special species might be used as potential markers for diagnosing and predicting colorectal adenoma. Similarly, it was confirmed that CRC-associated bacteria were changed with the degree of malignancy, and inflammatory factors (plasma C-reactive protein and soluble tumor necrosis factor II) increased across the adenoma-carcinoma sequence. However, there are still no absolute markers predicting the progression from adenoma to carcinoma. The findings from the current study will contribute to the development of the diagnostic biomarkers and therapeutic targets during the progression from adenoma to carcinoma.

Previous studies have reported that the composition and relative abundance of the intestinal microbiome would be influenced by age, gender, race, or dietary habits [20–24]. Our study has reached similar conclusions. Relative abundance of several bacterial species was altered between the different age and sex. Notably, Firmicutes dramatically decreased in the old patients compared to the young patients. Consistent with the previous studies, our results also demonstrated that the microbiome was different between the patients with the tumor in the left and right colon [9]. The relative abundance of *Bacteroides cellulosilyticus* was significantly increased with the order of differentiation degree in poor-moderate-well, and 9 CRC-associated bacterial species were significantly higher in the TNM stage III/IV group than in the TNM stage I/II group. The differences in the microbiota of patients with different tumor locations, differentiation degrees, and stages provide strong evidence of the tumor-host heterogeneity.

## 5. Conclusion

In conclusion, several intestinal bacteria changed along the adenoma-carcinoma sequence and might be the potential markers for the diagnosis and treatment of colorectal adenoma/carcinoma. Intestinal microbiota characteristics in CRC should account for the host factors.

## Figures and Tables

**Figure 1:** Intestinal microbiome richness and diversity in control, AD, and CRC groups. (a) Venn diagram illustrating the total, unique, and shared number of OTUs predicted for AD and CRC group datasets. (b) Rarefaction curve of OTU. (c) Species accumulation boxplot. (d) Boxplot based on Good's coverage. (e) Alpha diversity analysis based on the Chao1 index in AD and CRC groups (*P* = 0.95). (f) Alpha diversity analysis based on the Shannon index in AD and CRC groups (*P* = 0.74). (g) Principal coordinate analysis (PCoA) based on the weighted UniFrac distance matrix in AD and CRC groups (*Pr*(>*F*) = 0.33). (h) Nonmetric multidimensional scaling (NMDS) based on the weighted UniFrac distance matrix in AD and CRC groups (stress = 0.202). (i) Beta diversity analysis by the weighted UniFrac distance in AD and CRC groups (*P* = 0.88). (j) Principal coordinate analysis (PCoA) based on the weighted UniFrac distance matrix among control, AD, and CRC groups. (k) Nonmetric multidimensional scaling (NMDS) based on the weighted UniFrac distance matrix among control, AD, and CRC groups (stress = 0.123).

**Figure 2:** Top ten dominant genera in control, AD, and CRC groups.

**Figure 3:** Specific bacterial taxa associated with colorectal adenoma/carcinoma. (a) Venn diagram illustrating the total, unique, and shared number of significant pairwise difference at the genus level among control, AD, and CRC groups. (b) The relative abundance of the significantly changed genera among the three groups. (c) The most differentially abundant taxa between AD and CRC patients by linear discriminant analysis (LDA) effect size (LEfSe) analysis. Red bars indicate taxa enriched in the CRC group. (d) Microbial association network for colorectal adenoma/carcinoma-associated genera. (e) Receiver operating curve (ROC) by random forest analysis for distinguishing AD patients from CRC patients. (f) Mean Decrease Accuracy (MDA) coefficients of the 10 most important species in distinguishing AD patients from CRC patients. (g) Mean Decrease Gini (MDG) coefficients of the 10 most important species in distinguishing AD patients from CRC patients.

**Figure 4:** Association between fecal microbiota and CRC clinical characteristics: (a) the correlation heatmap between intestinal microbiota and age of CRC patients; (b) the correlation heatmap between intestinal microbiota and sex of CRC patients; (c) the correlation heatmap between intestinal microbiota and the tumor location; (d) the correlation heatmap between intestinal microbiota and the tumor stage.

**Table 1:** Demographic and clinical characteristics of patients and controls.

Characteristics	Control	AD	CRC
Number	199	20	154
Age (years)	59.48 ± 3.20	64.35 ± 12.89	65.81 ± 10.98
Sex			
Male	116 (58.29%)	15 (75%)	98 (63.64%)
Female	83 (41.71%)	5 (25%)	56 (36.36%)
Location^a^			
Left	—	19 (95%)	117 (75.97%)
Right	—	1 (5%)	37 (24.03%)
Size (mm)	—	—	4.55 ± 2.18
TNM stage^b^			
I	—	—	33
II	—	—	51
III	—	—	43
IV	—	—	10
NA	—	—	17
Differentiation degree			
Poor	—	—	9
Moderate	—	—	116
Well	—	—	9
NA	—	—	20
Pathological pattern			
Protrude	—	—	63
Ulcerative	—	—	69
NA	—	—	22
Histology			
Tubular	—	—	131
Mucinous	—	—	20
NA	—	—	3

CRC: colorectal cancer; AD: adenomas. ^a^The left colon was defined as the rectum, sigmoid, and descending colon; the right colon was defined as the transverse colon, ascending colon, and cecum. ^b^Tumor node metastasis (TNM) stage.

## Data Availability

The data used to support the findings of this study are included within the article.

## References

[1] Dekker E., Tanis P. J., Vleugels J. L. A., Kasi P. M., Wallace M. B. (2019). Colorectal cancer. *Lancet*.

[2] Bray F., Ferlay J., Soerjomataram I., Siegel R. L., Torre L. A., Jemal A. (2018). Global cancer statistics 2018: GLOBOCAN estimates of incidence and mortality worldwide for 36 cancers in 185 countries. *CA: a Cancer Journal for Clinicians*.

[3] Jeon J., Du M., Schoen R. E. (2018). Determining risk of colorectal cancer and starting age of screening based on lifestyle, environmental, and genetic factors. *Gastroenterology*.

[4] Tilg H., Adolph T. E., Gerner R. R., Moschen A. R. (2018). The intestinal microbiota in colorectal cancer. *Cancer Cell*.

[5] Zhang Y., Yu X., Yu E. (2018). Changes in gut microbiota and plasma inflammatory factors across the stages of colorectal tumorigenesis: a case-control study. *BMC Microbiology*.

[6] Feng Q., Liang S., Jia H. (2015). Gut microbiome development along the colorectal adenoma-carcinoma sequence. *Nature Communications*.

[7] Mizutani S., Yamada T., Yachida S. (2020). Significance of the gut microbiome in multistep colorectal carcinogenesis. *Cancer Science*.

[8] Xie Y. H., Gao Q. Y., Cai G. X. (2017). Fecal Clostridium symbiosum for noninvasive detection of early and advanced colorectal cancer: test and validation studies. *eBioMedicine*.

[9] Flemer B., Lynch D. B., Brown J. M. (2017). Tumour-associated and non-tumour-associated microbiota in colorectal cancer. *Gut*.

[10] Nakatsu G., Li X., Zhou H. (2015). Gut mucosal microbiome across stages of colorectal carcinogenesis. *Nature Communications*.

[11] Dai Z., Coker O. O., Nakatsu G. (2018). Multi-cohort analysis of colorectal cancer metagenome identified altered bacteria across populations and universal bacterial markers. *Microbiome*.

[12] Eckburg P. B., Bik E. M., Bernstein C. N. (2005). Diversity of the human intestinal microbial flora. *Science*.

[13] Wong S. H., Yu J. (2019). Gut microbiota in colorectal cancer: mechanisms of action and clinical applications. *Nature Reviews Gastroenterology & Hepatology*.

[14] Saus E., Iraola-Guzmán S., Willis J. R., Brunet-Vega A., Gabaldón T. (2019). Microbiome and colorectal cancer: roles in carcinogenesis and clinical potential. *Molecular Aspects of Medicine*.

[15] Ozato N., Saito S., Yamaguchi T. (2019). *Blautia* genus associated with visceral fat accumulation in adults 20 -76 years of age. *npj Biofilms and Microbiomes*.

[16] Warren R. L., Freeman D. J., Pleasance S. (2013). Co-occurrence of anaerobic bacteria in colorectal carcinomas. *Microbiome*.

[17] Flemer B., Warren R. D., Barrett M. P. (2018). The oral microbiota in colorectal cancer is distinctive and predictive. *Gut*.

[18] Jin H., Zhang C. (2020). High fat high calories diet (HFD) increase gut susceptibility to carcinogens by altering the gut microbial community. *Journal of Cancer*.

[19] Yuan L., Zhang S., Li H. (2018). The influence of gut microbiota dysbiosis to the efficacy of 5-fluorouracil treatment on colorectal cancer. *Biomedicine & Pharmacotherapy*.

[20] Delzenne N. M., Neyrinck A. M., Bäckhed F., Cani P. D. (2011). Targeting gut microbiota in obesity: effects of prebiotics and probiotics. *Nature Reviews Endocrinology*.

[21] Odamaki T., Bottacini F., Kato K. (2018). Genomic diversity and distribution of *Bifidobacterium longum* subsp. *longum* across the human lifespan. *Scientific Reports*.

[22] Ishibashi K. I., Nishioka M., Onaka N. (2019). Effects of Euglena gracilis EOD-1 ingestion on salivary IgA reactivity and health-related quality of life in humans. *Nutrients*.

[23] Nguyen S. G., Kim J., Guevarra R. B. (2016). Laminarin favorably modulates gut microbiota in mice fed a high-fat diet. *Food & Function*.

[24] Qi Y. F., Sun J. N., Ren L. F. (2019). Intestinal microbiota is altered in patients with gastric cancer from Shanxi Province, China. *Digestive Diseases and Sciences*.

